The article "Analysis of the Predictive Effect of Lactic Acid Combined with Cardiac Troponin T and 5-Hydroxytryptophan on the Severity of Sepsis in ICU Patients and Its Correlation with Prognosis" was retracted in 2023. Reasons: unreliable results or conclusions; lack of ethics approval or compliance; concerns about the data; concerns about the peer review.

# Analysis of the Predictive Effect of Lactic Acid Combined with Cardiac Troponin T and 5-Hydroxytryptophan on the Severity of Sepsis in ICU Patients and Its Correlation with Prognosis

**DOI:** 10.1155/2022/6215282

**Published:** 2022-09-16

**Authors:** Meini Jiang, Weidong Wu, Xiuzhe Wang, Caixia Zhao

**Affiliations:** ^1^Department of Intensive Care Unit, Shanxi Bethune Hospital, Shanxi Academy of Medical Sciences, Tongji Shanxi Hospital, Third Hospital of Shanxi Medical University, Taiyuan 030032, China; ^2^Tongji Hospital, Tongji Medical College, Huazhong University of Science and Technology, Wuhan 430030, China

## Abstract

In order to explore the effective markers of presepsis in the prediction of clinical disease and disease severity, the predictive effect of lactic acid (Lac) combined with cardiac troponin T (cTnT) and 5-hydroxytryptophan (5-HT) on the severity of sepsis in intensive care unit (ICU) patients and its correlation with prognosis is investigated. A total of 85 sepsis patients admitted to the ICU of our hospital from January 2020 to June 2021 are selected to establish the ICU sepsis group, and 72 health examination patients who received physical examination in our hospital during the same period are included in the healthy control group. The experimental results demonstrate that combined detection mode of serum Lac, cTnT, and 5-HT indicators has a high predictive value for the condition of patients with ICU sepsis and those indicators are closely correlated with the prognosis of patients. It suggests that the follow-up clinical monitoring of serum Lac, cTnT, and 5-HT indicators for patients with ICU sepsis can evaluate their condition and improve and optimize the clinical diagnosis and treatment plan effectively.

## 1. Introduction

Clinical studies have shown that the main cause of sepsis is severe infection and obvious systemic inflammatory reaction in patients. Without timely and effective treatment, patients are likely to delay the disease and cause further deterioration [1]. In severe cases, patients may have adverse symptoms, such as septic shock and multiple organ failure. This will seriously threaten the life and health of patients [2]. Therefore, early judgment and accurate evaluation of clinical sepsis can play a positive role in improving the prognosis and quality of life of patients [3]. Cardiac troponin T (cTnT) is a specific index of cardiac muscle. When the myocardium is damaged for various reasons, cTnT in the myocardium will be released into the blood and the concentration of cTnT in the blood will increase It is a very sensitive indicator. Slight myocardial injury will lead to the increase of cTnT in blood [4]. Cardiac troponin T has been used clinically as an important marker of acute and critical myocardial injury. The study found that this substance is abnormally overexpressed in patients with sepsis, indicating that the change of its content is closely related to the development and prognosis of the disease [5]. 5-hydroxytryptamine (5-HT) is a serotonin found in clinical research, which plays a certain role in the process of inflammation in the body. As a vasoconstrictor, 5-HT has been widely involved in physiological processes such as vascular function, hemostasis, liver regeneration, intestinal motility, insulin secretion, immune response, and so on. Some scholars have found in animal medical research that the abnormal expression of 5-HT in sepsis mice is one of the important risk factors leading to the decline of cardiac function [6]. As an intermediate product of glucose aerobic metabolism, lactate (Lac) can be significantly increased in oxygenation disorders and glucose anaerobic glycolysis. In sepsis, insufficient tissue perfusion can lead to a large accumulation of lac [7, 8]. It is worth noting that at present, no effective markers have been found in the prediction of clinical diseases and severity of sepsis. Therefore, the analysis of the application value of serum lac, cTnT, and 5-HT levels in ICU can provide clinical basis for the diagnosis and treatment of sepsis.

The article "Analysis of the Predictive Effect of Lactic Acid Combined with Cardiac Troponin T and 5-Hydroxytryptophan on the Severity of Sepsis in ICU Patients and Its Correlation with Prognosis" was retracted in 2023. Reasons: unreliable results or conclusions; lack of ethics approval or compliance; concerns about the data; concerns about the peer review.

The rest of this paper is organized as follows: Section 2 demonstrates the related work. Then, the proposed method and observation indicators are presented in Section 3.  Section 4 presents the comparative results and analysis.  Section 5 concludes the paper and gives the future work.

## 2. Related Work

Sepsis is a common clinical syndrome caused by infection. Relevant research shows that there are 18 million new cases of sepsis in the world every year. It has the characteristics of high clinical incidence rate, dangerous clinical symptoms, and high mortality [9]. The pathogenesis is that the bacteria and infected foci caused by the infection in the patient have an adverse effect on the balance of local blood circulation, which makes the microcirculation function of relevant tissues disordered in the process of disease, thus affecting the patient's heart and other organs. This will lead to myocardial cell damage and insufficient heart filling, imbalance of oxygen supply, and demand in tissues and organs [10, 11]. In recent years, medical institutions have carried out a large number of clinical studies on the treatment of sepsis. Relevant antiinfection treatment schemes have been continuously improved, and the level of clinical medical technology has also been continuously improved. However, clinical data show that the mortality control of sepsis has not achieved the expected effect, which poses a great threat to human health. Therefore, it is of great significance for the early diagnosis and prognosis of sepsis [12].

The article "Analysis of the Predictive Effect of Lactic Acid Combined with Cardiac Troponin T and 5-Hydroxytryptophan on the Severity of Sepsis in ICU Patients and Its Correlation with Prognosis" was retracted in 2023. Reasons: unreliable results or conclusions; lack of ethics approval or compliance; concerns about the data; concerns about the peer review.

The clinical symptoms of sepsis are not specific, and its clinical diagnosis and severity assessment are still very difficult. When sepsis occurs, the relevant laboratory indicators in patients will show abnormal expression, and the measurement of biomarkers in sepsis can provide reference for clinical treatment decisions and prognosis of sepsis [13]. The results show that compared with healthy people, serum lac, cTnT, and 5-HT are higher in ICU sepsis patients, confirming that the abovementioned three indicators are abnormally high after the onset of sepsis. As the intermediate product of glucose aerobic metabolism and the end product of anaerobic metabolism, lac can be used to measure whether the metabolism is in an anoxic state. Moreover, the kidney has abundant blood flow and is extremely sensitive to tissue ischemia. In sepsis patients, tissue ischemia and hypoxia will lead to lac aggregation and abnormally high expression, suggesting that this indicator may be closely related to the prognosis of patients [14]. In addition, previous studies have confirmed that the cardiac cell membrane is more complete in the normal state of the body, so cTnT substances are difficult to enter the cell membrane and participate in the blood circulation, so the cTnT expression in the plasma of healthy people is low. When myocardial cell injury occurs, the cell membrane rupture leads to the troponin complex released from the myocardium into the blood, resulting in the high expression of cTnT in patients with sepsis, which also suggests that the abnormally high expression of cTnT is an important manifestation of impaired myocardial function and may have adverse effects on the prognosis of patients with sepsis [15, 16]. As a biogenic amine derivative, 5-HT is not easy to cross the blood-brain barrier and has different distribution and functions in different parts of the human body. Studies have found that the 5-HT receptor is expressed in human immune cells, including neutrophils, macrophages, and dendritic cells [17]. The results showed that the serum 5-HT increased significantly in patients with sepsis. In the early stage of sepsis, microorganisms can invade the body, macrophages and neutrophils can move to the inflammatory site, and increase free radicals, promoting oxidative stress response. Studies have shown that septic mice have obvious oxidative stress response, and the oxidative stress of the liver, kidney, and other tissues of mice with low 5-HT level is significantly reduced [18, 19]. This suggests that 5-HT may aggravate sepsis by promoting inflammatory and oxidative stress responses. Relevant results confirmed that the combination of serum lac, cTnT, and 5-HT can better predict the prognosis of the disease, suggesting that in the treatment of sepsis, it is necessary to guard against the occurrence of myocardial damage in such patients, pay attention to the treatment of sepsis patients with serum lac, cTnT, and 5-HT, and pay attention to myocardial protection, so as to reduce the mortality of patients with sepsis [20]. In addition, the comprehensive use of different biomarkers can improve the ability to judge the prognosis of sepsis, which provides certain guidance for clinical treatment [21, 22].

The article "Analysis of the Predictive Effect of Lactic Acid Combined with Cardiac Troponin T and 5-Hydroxytryptophan on the Severity of Sepsis in ICU Patients and Its Correlation with Prognosis" was retracted in 2023. Reasons: unreliable results or conclusions; lack of ethics approval or compliance; concerns about the data; concerns about the peer review.

## 3. Proposed Method and Observation Indicators

### 3.1. General Information

A total of 85 sepsis patients admitted to the intensive care unit (ICU) of our hospital from January 2020 to June 2021 are selected to establish the ICU sepsis group, and a total of 72 health examiners who received physical examination in our hospital during the same period are included in the healthy control group. In the ICU sepsis group, there are 44 males and 41 females, aged 36–68 years, with an average of (50.65 ± 10.38) years, and body mass index (BMI) ranged from 16.94 to 26.07 kg/m^2^, with an average of (21.35 ± 2.50) kg/m^2^. In the healthy control group, there are 39 males and 33 females, aged from 34 to 70 years old, with an average of (50.44 ± 10.34) years old. BMI ranged from 17.12 to 25.96 kg/m^2^, with an average of (21.41 ± 2.54) kg/m^2^. The baseline data include the comparison of gender, age, and BMI, *p* > 0.05, which confirms that the comparison between the two groups is scientific and reasonable. The prognosis of patients with sepsis in ICU is analyzed and related data are collected. According to the prognosis, subgroups are established for patients with sepsis in ICU, including the better prognosis group and the poor prognosis group.

Inclusion criteria for patients with sepsis in ICU are as follows: (1) Clinical symptoms and related diagnostic results of patients are in line with the relevant diagnostic criteria in sepsis prevention and treatment. (2) Clinicopathological and previous medical history of the patients are complete. (3) Patients are not complicated with serious neurological diseases and could be assessed by the acute physiological and health-related scales in our hospital. (4) Patients with high clinical compliance can cooperate to participate in the follow-up investigation related until the end of the study.

ICU sepsis patients' exclusion criteria are as follows: (1) Patients complicated with the liver, kidney, and other serious organic dysfunction diseases. (2) Patients complicated with malignant tumor disease or serious cardiovascular and cerebrovascular diseases. (3) The patient has severe coagulation dysfunction in the blood system. (4) Women in pregnancy/lactation.

The article "Analysis of the Predictive Effect of Lactic Acid Combined with Cardiac Troponin T and 5-Hydroxytryptophan on the Severity of Sepsis in ICU Patients and Its Correlation with Prognosis" was retracted in 2023. Reasons: unreliable results or conclusions; lack of ethics approval or compliance; concerns about the data; concerns about the peer review.

### 3.2. Index Detection Method

All subjects in this study agreed and accepted serum lac, cTnT, and 5-HT detection. Among them, the ICU sepsis group is tested within 24 h after admission for diagnosis and the healthy control group is tested on an empty stomach in the morning of physical examination. 8 mL peripheral elbow venous blood is extracted from all subjects, followed by a centrifugation operation with parameters set at 3500 r/min, centrifuge radius of 10 cm, and centrifugation duration of 15 min. After the operation, the supernatant is taken for testing. cTnT shall be determined by a Danish AQT90 FLEX analyzer within 6 h, during which relevant reagents shall be applied and corresponding operations shall be completed in strict accordance with relevant instructions of reagents. The serum lac level is detected by an automatic blood gas analyzer. Serum 5-HT is determined by liquid chromatography and an Orbi Trap EXploris480 high resolution mass spectrometer.

### 3.3. Observation Indicators

The observation indicators mainly include the following: (1) Serum lac, cTnT, and 5-HT levels are compared; (2) the ROC curve is used to analyze the predictive efficacy of single indicators of serum lac, cTnT, and 5-HT and combined detection modes for sepsis; (3) the serum lac, cTnT, and 5-HT levels of patients with different prognosis in ICU sepsis group are compared; and (4) to analyze the correlation between serum lac, cTnT, and 5-HT expression and prognosis of ICU patients with sepsis.

### 3.4. Statistical Processing

SPSS 26.0 software is used for statistical analysis of the data involved in this study, and the measurement data are verified. Mean ± standard deviation ($\bar{x}$ ± *s*) is used to represent the data differences between groups and *t* test is performed. The count data involved are represented by (*n*, %), and the data differences between groups are analyzed by *χ*^2^ test. Spearman correlation coefficient is used to analyze the correlation between the prognosis of ICU patients with sepsis and serum lac, cTnT, 5-HT. In this study, the prediction and diagnostic value evaluation of sepsis are completed by the ROC curve, and *p* < 0.05 syndrome data are statistically different.

## 4. Comparative Results and Analysis

### 4.1. Serum Lac, cTnT, and 5-HT Levels Are Compared

Serum lac, cTnT, and 5-HT indexes in ICU sepsis group increased significantly than the healthy control group (*p* < 0.05) as shown in Table 1.

The article "Analysis of the Predictive Effect of Lactic Acid Combined with Cardiac Troponin T and 5-Hydroxytryptophan on the Severity of Sepsis in ICU Patients and Its Correlation with Prognosis" was retracted in 2023. Reasons: unreliable results or conclusions; lack of ethics approval or compliance; concerns about the data; concerns about the peer review.

### 4.2. ROC Curve Is Used to Analyze the Predictive Efficacy of Single Indicators of Serum Lac, cTnT, and 5-HT and Combined Detection Modes for Sepsis

The ROC curve is used to analyze the low detection efficiency of single indicators of serum lac, cTnT, and 5-HT, and the prediction efficiency of the three combined modes increased significantly than that of single detection mode (AUC = 0.960) as shown in Table 2 and Figure 1. The results show that the diagnostic efficiency of single indicator is low, and the efficiency of the three combined detection is high.

### 4.3. Serum Lac, cTnT, and 5-HT Levels of Patients with Different Prognosis of ICU Sepsis

According to the prognosis of patients in the ICU sepsis group, subgroups are established, including the better prognosis group (*n* = 54) and the poor prognosis group (*n* = 31). The serum indexes of lac, cTnT, and 5-HT in the poor prognosis group increased significantly than those in the better prognosis group (*p* < 0.05) as shown in Table 3.

### 4.4. Analysis of the Correlation between Serum Lac, cTnT, and 5-HT Expressions and Prognosis of ICU Patients with Sepsis

Spearman correlation coefficient analysis showed that serum lac, cTnT, and 5-HT expressions are significantly positively correlated with poor prognosis in ICU patients with sepsis (all *p* < 0.05) as shown in Table 4. The comparative analysis of patients with different prognosis showed that the serum indicators of patients with poor prognosis are significantly higher than those of patients with better prognosis. In addition, the prognosis of patients with ICU sepsis is significantly positively correlated with serum lac, cTnT, and 5-HT, which is basically consistent with the previous studies.

## 5. Conclusions

In this study, the effective markers of presepsis in the prediction of clinical disease and disease severity are explored and the predictive effect of lactic acid combined with cardiac troponin T and 5-hydroxytryptophan on the severity of sepsis in intensive care unit patients and its correlation with prognosis is investigated. From the experimental results, serum lac, cTnT, and 5-HT are highly expressed in ICU sepsis patients. Combined monitoring of the three indicators has important effects on early diagnosis, and prognosis of ICU sepsis patients. Dynamic monitoring of the three indicators can be carried out in subsequent clinical practice to optimize and improve the clinical diagnosis and treatment plan. It has positive effect on improving the prognosis of patients with sepsis. However, this study may have some limitations, especially about all the enrolled cases are surgical patients and the number is insufficient. In the future research, we will expand the scope and number of cases to verify the results of this study.

The article "Analysis of the Predictive Effect of Lactic Acid Combined with Cardiac Troponin T and 5-Hydroxytryptophan on the Severity of Sepsis in ICU Patients and Its Correlation with Prognosis" was retracted in 2023. Reasons: unreliable results or conclusions; lack of ethics approval or compliance; concerns about the data; concerns about the peer review.

## Figures and Tables

**Figure 1:** ROC chart of serum lac, cTnT, and 5-HT for single and combined detection of sepsis.

**Table 1:** Comparison of serum lac, cTnT, and 5-HT levels ($\bar{x}$ ± *s*).

Group	Lac (mmol/L)	cTnT (ng/mL)	5-HT (*μ*mol/L)
ICU sepsis group (*n* = 85)	2.34 ± 0.37	0.28 ± 0.05	2.33 ± 0.20
Healthy control group (*n* = 72)	1.45 ± 0.23	0.19 ± 0.03	1.84 ± 0.14
*t*	17.712	13.367	17.473
*p*	<0.001	<0.001	<0.001

**Table 2:** Predictive efficacy of lac, cTnT, and 5-HT single indicators and combined detection modes for sepsis.

Indicators	AUC (95%CI)	Sensitivity (%)	Specificity (%)	About an index	Cutoff value
Lac (mmol/L)	0.772 (0.697∼0.847)	78.00	77.50	55.50	2.15
cTnT (ng/mL)	0.779 (0.706∼0.852)	80.00	78.00	58.00	0.24
5-HT (*μ*mol/L)	0.615 (0.525∼0.705)	72.00	74.50	46.50	2.07
Union	0.960 (0.933∼0.987)	86.00	92.50	78.50	—

**Table 3:** Comparison of serum lac, cTnT, and 5-HT in ICU patients with different prognosis ($\bar{x}$ ± *s*).

Group	Lac (mmol/L)	cTnT (ng/mL)	5-HT (*μ*mol/L)
Group with better prognosis (*n* = 54)	2.12 ± 0.27	0.25 ± 0.03	2.21 ± 0.14
Poor prognosis group (*n* = 31)	2.72 ± 0.11	0.33 ± 0.02	2.54 ± 0.58
*t*	−11.799	−13.238	−3.999
*p*	<0.001	<0.001	<0.001

**Table 4:** Correlation analysis between serum lac, cTnT, and 5-HT expression and poor prognosis of ICU sepsis.

	*Patients with sepsis in ICU have a poor prognosis*	
	*Rs*	*p*
Lac (mmol/L)	0.833	<0.001
cTnT (ng/mL)	0.832	<0.001
5-HT (*μ*mol/L)	0.834	<0.001

## Data Availability

The simulation experiment data used to support the findings of this study are available from the corresponding author upon request.
